# An Evaluation of Human Conversational Preferences in Social Human-Robot Interaction

**DOI:** 10.1155/2021/3648479

**Published:** 2021-02-22

**Authors:** Chapa Sirithunge, A. G. Buddhika P. Jayasekara, D. P. Chandima

**Affiliations:** Intelligent Service Robotics Group, Department of Electrical Engineering, University of Moratuwa, Moratuwa 10400, Sri Lanka

## Abstract

To generate context-aware behaviors in robots, robots are required to have a careful evaluation of its encounters with humans. Unwrapping emotional hints in observable cues in an encounter will improve a robot's etiquettes in a social encounter. This article presents an extended human study conducted to examine how several factors in an encounter influence a person's preferences upon an interaction at a particular moment. We analyzed the nature of conversation preferred by a user considering the type of conversation a robot could have with its user, having the interaction initiated by the robot itself. We took an effort to explore how such preferences differ as the factors present in the surrounding alter. A social robot equipped with the capability to initiate a conversation is deployed to conduct the study by means of a wizard-of-oz (WoZ) experiment. During this study, conversational preferences of users could vary from “no interaction at all” to a “long conversation.” We changed three factors in an encounter which can be different from each other in each circumstance: the audience or outsiders in the environment, user's task, and the domestic area in which the interaction takes place. Conversational preferences of users within the abovementioned conditions were analyzed in a later stage, and critical observations are highlighted. Finally, implications that could be helpful in shaping future social human-robot encounters were derived from the analysis of the results.

## 1. Introduction

Acceptance of service robots in social environments has inspired many researchers to explore human tendencies when dealing with social robots. Conventional service robots deployed in social environments are expected to support daily routine tasks such as cooking, cleaning, and taking care of health [1–3], but modern assistive robots must also have cognitive skills to maintain a friendly and human-like interaction with the humans they daily meet [4]. For these robots, to be accepted by its user for a long duration, certain human-like qualities have to be embedded. Perceived sociability, cognitive skills, and adaptation are found to be the key factors considered in long-term acceptance of a social robot [5]. Furthermore, making right interaction decisions is equally important in playing the role of a companion rather than being just a service provider [6, 7]. These features ease dealing with the robot without stressing out its user with a set of restrictions to abide by during an interaction with the robot.

Intelligence in initiating conversations at right occasions is highly appreciated in achieving a robot's context-aware behavior. Many users prefer to interact with robots, with speech [8], and the nature of speech must be friendlier and human-like. In other words, these robots are preferred to determine when to interact and when not to. During the interaction, this natural behavior enhances the cohesion between robot and its nonexpert user. Such robotic systems which can replicate complex human behavior in order to play the role of a close contact such as “friend” rather than a “servant” are being developed [9–13]. On the one hand, humans prefer robots with at least some context awareness as well, in addition to performing a predefined set of tasks. As a result, robots can collaborate with people without disturbing them when they are engaged in an activity. On the other hand, when robots have an instinct of how to co-op with the situation, users do not need to stress themselves with a set of predefined behaviors that are perceivable by the robot. Therefore, robotic systems, which adapt to the circumstances in a certain encounter, are demanding in this era. Hence, social intelligence is an emerging requirement in human-robot interaction concerning social environments.

Likeliness of the robot being accepted as a conversational partner depends on the environment as well as the current task of the user. The study in [14] ensures how the social behavior of a robot improves the acceptance from its users as a companion in social human-robot domains. We investigate how the nature of interaction initiated by the robot affects its acceptance by a human. Subsequently, a set of affect-based types of conversation were selected and implemented on a service robot in a simulated social environment in which few users were present or only a single user was present. This study is intended to find human tendencies towards interaction in different situations and hence will provide means of engraving social skills into a robot's behavior before utilizing in human environments. To support this approach, we conducted a wizard-of-oz study to explore the nature of human conversation with the presence of a service robot when several factors in the environment vary. Factors which are more likely to have an influence upon the conversational preference of humans are selected. The type of interaction preferred by the user was used as a mediator to perceive user situation and the level of interest towards the interaction initiated by the robot. Responses observed during the study can be used to upgrade existing robots' perception of human behavior. Hence, this will allow a robot to be a successful companion to the human without violating user expectations.

As humans establish emotional ties with whom they interact, this fact may remain the same for a human-robot interaction as well. Hence, the proactive, social means of engagement are expected from a robot in such a scenario [15]. One aspect in developing mechanisms to enhance social intelligence in robots is to improve the user experience with such robots. A similar study was conducted to analyze conversational preferences of schizophrenia patients with robots in [16]. Even so, only the context covers only patient-robot interaction, not human-robot interaction entirely.

According to the survey by Lorenza et al. [17], the cognitive, emotional, and behavioral examination of human responses have an impact upon a robot's behavior. Therefore, to measure this impact adequately beforehand, it is important for the robots to be cautious upon the factors which affect a human's interaction decisions during a particular encounter. From this study, we intend to lay a justifiable basis to bring several such observable factors that can be used by a robot to evaluate an encounter before robot-initiated interaction. We considered observable cues from humans as well as their surroundings, which were likely to have an impact towards responses generated by a human in a certain instance.

## 2. Related Work

In order to participate in collaborations with people, robots must not only see and talk with people but also make use of the conventions of conversation to connect with their human counterparts. In [18], the authors have investigated occasions in which active collaboration between a robot and a human is required in service applications. Perceived connection between the human and the robot becomes effective, and the mutual interest grows when the two participants can understand the intentions of each other in a conversation; for instance, when to continue interaction and when to stop. As per this study, understanding the situation of a human is a demanding feature in robot's acceptance within a sociable human environment.

Certain features and behaviors embodied in robots make an impact on people's willingness to engage in at least a short interaction with the robot. The work explained in [19] has presented a set of social rules for robot behavior (a “robotiquette”) that is comfortable and acceptable to humans. According to that, the conceptual space of HRI (human-robot interaction) studies expects a robot companion in a home environment to “do the right things” and “fulfil its tasks” in a manner that is acceptable and comfortable to humans. Furthermore, real-time performance of the robot which follows human social conventions and norms is more likely to be accepted for a long duration by humans [20].

In [21], a robot which is also an intelligent weight loss coach has been implemented. This makes an excellent example for the situation perception embodied in the robot itself and hence has been exploited to reduce obesity. During this case, results show that the robot is accepted for a long-term interaction by its users. However, this robot is not fully capable to identify user behaviors which are not related to physical health. But the fact that a higher social intelligence as well as a greater acceptance from the user can be achieved by engraving abilities related to emotional and instinctive behavior cannot be neglected in this scope [22]. Furthermore, there are many robotic systems to carry out a smooth conversation but the capability of these systems is limited to only after the initiation of a conversation but not before the conversation [23]. In [24], conversation was used as a part of assistance for Alzheimer patients in addition to therapy. This study has identified robot's knowledge of the location, patient's history, type of disease, etc. and these parameters are important to decide the level of interaction between the patient and the robot.

Law et al. [25] present a similar approach towards understanding one aspect in this regard. The authors have conducted a human study by means of a wizard-of-oz experiment, to assess the level of curiosity aroused in humans when dealing with an assistive robot. Study confirmed the fact that the human curiosity considerably changes when the intelligence of the robot is higher. Moreover, it is found that the social acceptance of a service robot increases when a robot is able to perceive the very needs of a user and act accordingly [26]. Results of the human study in [27] verify that humans prefer user adaptive dialogs in conversations even with a robot. The work explained in [28] is a promising example of the growing rapport between humans and robots with such an intelligence. Human further prefers the companionship build through interactive conversation between him and the robot; in addition to the service purposes, most robots are intended for [29].

A method for attention estimation is proposed in [30]. Authors have used human pose and speeds of specific angular joints to identify the nonverbal interaction demanding of a user. These two parameters were evaluated using a fuzzy logic-based mechanism to evaluate the interest level of a human towards a robot. However, these are not the only parameters which define the nonverbal interaction demanding of a human. According to a review assessment performed in [31], wizard-of-oz is an effective mechanism to study human tendencies based on nonverbal behavior. WoZ studies are effective in assessing such interactive sessions in a short period without unnecessary preparations beforehand. An example scenario which evaluates speech-based interactive interfaces is presented in [32]. In [33], Sidner et al. further elaborate that the dialog features are important in accepting a robot for a long duration during human-robot interaction.

The above discussed systems access a limited number of cues from its users and their surroundings before making interactive decisions. Still, there are several other factors to be considered before generating responses in a human-robot social encounter [34]. We selected several such factors which are likely to have an impact upon user responses during an encounter and investigated whether these factors actually make such an impact. Hence, the findings of the study can be used to improve the conceptual basis of reasoning in future social robots.

In our work, the importance of understanding user situation is evaluated using such a WoZ approach. Factors used to define user situation were the activity or the current task of the user, number of people around the user, and the type of area of the house. Conversational preferences when these factors change were analyzed with the help of a domestic service robot platform placed in a simulated social environment.

Since our work is based on verbal human behavior, a WoZ experiment will have the capability to explore unexpected tendencies in human behavior prior to an interaction. In this work, we tried to investigate human behaviors that can be used as cues for a robot to perceive user situation prior to an interaction. It is expected that these findings will help improve social intelligence of a social robot for the purpose of caretaking and simultaneously providing emotional support through interaction.

## 3. Theoretical Approach

### 3.1. Robot's Perception of the Environment

A situation between a human and a robot consists of the *robot* itself, the *user* (human), and the *environment* (objects and space) around the robot and the user. When the robot intends to perceive such a situation, it first has to identify interactive factors within itself, the environment, and the user. Factors within the robot itself include the dialog patterns the robot generates, maintaining an interactive distance in between, and displaying appropriate behavior, etc. Factors within the user will be numerous, but emotions, social norms, beliefs, personality traits, user's activity at that moment, and other psychophysiological factors contribute majorly in deciding the level of interaction readiness within a human. Objects and other humans in the surrounding, obstacles, etc. make the list of factors in the environment which have to be perceived by the robot.  Figure 1 demonstrates this idea.

### 3.2. Theory of Planned Behavior

Out of many psychological theories behind human tendencies, theory of planned behavior lays a reasonable, yet justifiable basis for the differences in human behavior under various circumstances in the environment.

According to the theory, one's believes are linked to his/her behavior. This makes reasoned actions based on a restricted or controlled behavior. An individual's intention of a certain behavior at a specific time, a place, etc. is based on the regulations that humans follow by. These will take three forms: behavioral, normative, and control. The theory of planned behavior comprises of six constructs that collectively present actual control of a person over the behavior [35]. These constructs are stated briefly as follows.

1. Attitudes—degree to which the individual has a favorable or an unfavorable evaluation upon the behavior of interest
2. Behavioral intention—motivational factors that influence the behavior
3. Subjective norms—belief about whether behavior will be approved by peers and people of importance
4. Social norms—customary behavior in a group of people belonging to a cultural context
5. Perceived power—the behavioral control over these factors that may facilitate or impede performance
6. Perceived behavioral control—person's perception of ease or the difficulty in performing the action

This concept can be related to human-robot scenario as follows. Due to the factors in the environment, user's perception of the environment or the surrounding may subject to change, depending on his/her beliefs. Hence, the reaction towards robot's conversations may change in different scenarios. Three factors which are most likely to affect the user response are considered in this study. These factors are selected from *user* and *environment* aspects. The purpose of this is to evaluate the human behavior during these situations. These factors are listed below.

- Task of the user—e.g., having a snack, cleaning, and engaged in a desk activity
- People in the surrounding—alone or surrounded by few people
- Type of area in the domestic/social environment—living room, bed room, or kitchen

These three factors contribute to evaluate mainly attitudes, subjective norms, and perceived behavioral control out of the six constructs of the theory of controlled behavior. It is assumed that the type of interaction preferred by the user change when these factors change. We evaluated this fact through the human study conducted in the form of the WoZ experiment.

An application of the two theories: occasion 1 (a), user was working and has no idea about the presence of the robot, (b) notices the presence of the robot as it moves and as a result, the user looks at the robot, and (c) stops the work and gives attention to the robot while it approaches the user.

An application of the two theories: occasion 2 (a), user was working and has no idea about the presence of the robot, (b) notices the presence of the robot as it moves and looks at the robot, (c) user averts her gaze and give attention to the work, and (d) engage in the work again.

### 3.3. Theory of Reasoned Action

The theory explains that there is a relationship between one's attitudes and actions [36]. Hence, the theory is used to predict the behavior of a human in a particular scenario, based on the preexisted attitudes and behavioral intentions of that individual. That individual's expectations upon the outcomes of a behavior controls his/her decision to adopt that behavior. This fact is deployed in exploring the tendencies in human behavior in the presence of the robot used in the WoZ study. In such a situation, there are few stages which a user goes through; for instance, noticing the presence of the robot, responding towards robot which approaches towards him/her, initiating a conversation with the robot, or responding to a conversation initiated by the robot can be stated as the usual stages of interaction in such a situation. The user's conversational preferences might change according to his/her attitudes, beliefs, and expectations in such an instance. These attitudes, beliefs, and expectations may subject to change depending on the factors present in the environment, and this fact is going to be evaluated through this study.

Example scenarios encountered in a social environment with the presence of humans and robots as perceived by the above theories are given in Figures 2 and 3. In occasion 1 (Figure 2), the user gave priority to an interaction with the robot, but in occasion 2 (Figure 3), the user gave priority to her current activity. In both the occasions, various factors within the environment and the user itself will affect her response.

## 4. Experiment

### 4.1. Setting and the Research Platform

The experiment was conducted in a simulated social environment in the laboratory. Participants were students, nonacademic staff members of the university, and some outsiders in the age range 19-58 (Mean-28.45, SD-9.02) who volunteered the study. There were 37 participants, and they were in good health condition without any physical defects which will alter their reactions during the study. More than half of the participants did not have a technical background in education, majors, or research related to Engineering. The gender of the user was not included within the scope of this study. Upon arrival, the users were given instructions regarding the tasks they should complete but they were not aware of the fact that they are intended to talk to the robot but they are instructed to respond towards the robot if the robot initiates an interaction. They were not knowledgeable about the exact intention of the experiment because that will cause a bias response from users towards the robot. Hence, the participants were instructed to perform a given activity in the way they are used to perform that before.

The experiment was conducted using a service robot called MIRob. The robot is visually and verbally capable and has the ability to approach a user, make a conversation, and handle objects. This is a Pioneer 3DX MobileRobots platform equipped with a Cyton Gamma 300 manipulator and a Kinect camera for vision. The maps required to navigate around were created with Mapper3 Basic software. The platform is equipped with a microphone and a speaker to listen to and respond its users. This platform is shown in Figure 4.

### 4.2. Procedure

The selected user was allowed to engage in a certain task, and the robot was allowed to approach the user to initiate a conversation with him/her. The user was advised to complete a certain task and if the robot talks to him/her, to talk back. The set of tasks to be performed by the users was predefined. There were separate lists of tasks to be performed in the living room, bed room, and kitchen. The participant or the user was knowledgeable on the tasks that are to be performed in each living area. The tasks were selected so that there will be at least three tasks performed in each area. These tasks are the most common to that particular social or domestic environment, and few tasks selected for the study are listed in Table 1. While the user was engaged in a task, the robot was remotely guided towards him/her and was allowed to initiate an interaction in the ways given below. This set of experiments was conducted over a period of 7 days, so that the participants had enough time in between tasks. This prevented participants getting exhausted and hence generating biased, involuntary responses towards the robot. People in the surrounding were not participants but one or two members from the set of experimenters. And all 37 users participated in the experiments at least for three different tasks. As the number of participants was 37, each conducted 12 tasks, 2 times (alone and with the presence of a few others in the surrounding), the experiment was conducted 888 times throughout a week. We kept gaps in between experiments to avoid users repeating the same response over and over by practice. The map of the environment was predefined in the simulation. Therefore, the robot navigated to the target positions and its orientation which were defined by the operator. In this scenario, the target position of the robot was a point within the interactive area near the user. For the ease of future referencing, these types of conversational preferences are abbreviated as follows.

NI-No interaction

GRT-Greeting

SER-Asking to deliver a service

TLK-Small talk

CON-Long conversation.

How a conversation is categorized into these types is shown in Figure 5. As the conversation extends, the type of conversation shifts from NI to a CON. The robot will not talk to its user during NI. In GR, the robot will only greet the person and navigate away. The greeting will just be a single sentence saying “good morning,” “hey,” “hello,” etc. In SER, the robot will ask to deliver something for the user, as an assistance to his/her current task. This will be approximately four sentences maximum in the entire conversation. In the TLK, the robot will say a few additional sentences other than greeting and sometimes will ask if the user wants something. Such a conversation consisted of about 5-7 sentences. All the conversations longer than that were considered as CON. Such conversations cover a broader scope of topics as well as these existed for a longer duration. Therefore, the duration of the conversation depended on the type of conversation robot had with a user. In all the occasions, the robot stopped continuing the conversation depending on the curiosity of the user to engage with the robot or when the conversation seems to disturb the user. During the experiment, robot had a CON with its user and in the end, a survey was conducted to know the actual preference of the user. Users were shown how the type of conversations are categorized and were asked to select their preference at a similar occasion in the participant's own domestic environment despite the conversation he/she already had with the robot.

The robot initiated a conversation despite the task of the user, and user responses towards that interaction were recorded. Voice responses were monitored remotely by an operator without the knowledge of the user. Furthermore, a single participant was asked to perform all the tasks listed in the experiment separately in different occasions. Each task was performed twice: when the user was alone and when few others are present. The second occasion replicates a typical domestic or a social environment in which family members or few other known persons are present around. In the experiment, participants in a single setting were acquaintances. For instance, if there were few people around the user at the time of the conversation, all these people were acquaintances but were not related to each other.

MIRob was remotely controlled by a human operator. Robot responses were generated with respect to the user response in each occasion. It is expected to assess the effect of considered factors in the surrounding upon human conversational preferences, in both qualitative and quantitative manners. Therefore, the independent variables used in the study were the task, area of the social environment (living room, bedroom, or kitchen), and whether few people were present around the user or not. The type of interaction preferred by the user is used as the dependent variable in the analysis stage. As stated earlier, in the experiment, the same occasion was analyzed under two categories: when only the user was present and when there were few other people were around. An important fact to be considered in this case was that when few other people were present around, they were not involved in the interaction process except when the user was having a conversation with them. As the experiment was conducted by means of a WoZ, the robot operator monitored the robot towards a point closer to the user. Voice responses were generated after the robot approached the user. Path planning and navigation of the robot were autonomous while tracking of the user and generation of voice responses were teleoperated by the human operator. Therefore, the operator instructed the robot where to approach and what to speak. None of the persons in the environment participated in the conversation with the robot except the intended participant.

As MIRob was monitored by a human operator, its voice responses were generated in accordance with the responses from the participant. The responses of the robot during the experiment include only maintaining a socially interactive distance between the robot and the user and voice. If any of the users does not respond the robot, the robot was instructed to leave without causing any distraction. In such a situation, the robot assumes that the user does not prefer to interact.

Independent variables used in the experiment were the task of the user, domestic area, and the presence of others in the surrounding. The conversational preference was the dependent variable during analysis. The assumption made during the study was that there is no significant difference between the groups used for comparison purposes.

### 4.3. Results of the Experiment

After the experiment, the conversational preferences of users were analyzed using statistical methods. The first question of interest was whether there is a difference in user responses depending on the number of people in the surrounding.  Table 2 shows a comparison of the percentage frequency of each type of interaction for the two occasions: when the user was alone and when few people were around. This study was intended for all the tasks listed in Table 1. As seen from the results, there is an increase in demanding a service or limiting the conversation just for a greeting when few other people were present in the surrounding. As seen from this information, the demand for interaction types NI, GRT, and SER have been increased by 15% when the number of people around the user has increased from zero to a few. In the same way, the tendency towards friendly conversations (TLK and CON) has been reduced from 36% to 21%, i. e., by 15%. In this case, types of interactions NI, GRT, and SER are categorized into a single group for analysis because these types are preferred by humans in official situations and whenever there is little time for relaxation or friendly behavior. Therefore, TLK and CON, which fall under friendlier conversational preferences, are grouped together. An example scenario from the experiment is given in Figure 6 when the user was alone. A scenario when there were people around is shown in Figure 7. In this situation, the user preferred a long conversation when she was alone, and a service when there was a second person in the kitchen. Such behavioral changes were recorded during the experiment.

Table 3 shows an ANOVA test performed on the same data for the comparison of percentage frequencies of each type of conversational preference in each area of the social environment. The test was performed to analyze how the tendency towards each type of conversational preference changes when the domestic area changes. Here, living room, bed room, and the kitchen were used as living areas as mentioned before. Percentage usage of the types of interaction is calculated and compared. First, test was implemented for the case when only the user was alone in the considered environment, and the second test for the case when few others were present in the surrounding, in addition to the user. From the test, it was intended to find the differences in conversational preferences when condition of the surrounding with regard to the peer (whether the user was alone or there were few others around) was kept constant. Furthermore, it was expected to find whether there is a change in user behavior upon where the user is, despite whether he/she is alone or with few people around.

Table 4 shows the results of a *t*-test performed to test the deviation between the preference of each type of interaction when alone and when surrounded by a few. Changes in demand for each type of interaction in the said two occasions were analyzed without an involvement of other types of conversational preferences. Frequency of the type of interaction in each domestic area was taken as data for the *t*-test. This explored unexpected tendencies in human behavior, and an in-depth analysis of the results is given in the discussion.

Shown in Table 5 are two ANOVA tests performed on the same set of data to test the deviation between the conversational preferences during the list of selected tasks while the user was alone and with one/few people around. The frequency of using each conversational preference during these tasks was calculated and analyzed for the deviations between each group. Here, the groups were the conversational preferences from NI to CON and the frequencies were listed according to the tasks listed in Table 1. In both the situations in Table 5, when alone and when surrounded by few people, the *F* critical value was 2.539.

### 4.4. Observations and Discussion

From the results displayed in Table 2, demand for conversational preferences NI, GRT, and SER was decreased by 15% as the number of people around the user changed from “none” to “few.” It can be seen that the tendency of the user towards a friendly interaction reduced when there were people around. Even though these people were not directly involved with him/her, their presence influenced the reactions of the user towards robot. This could be explained using the theory of planned behavior [37]. A perceived behavioral control could be observed within the user due to such changes in the surrounding.

Most important and unexpected patterns in user behavior were demonstrated from the *t*-test shown in Table 4. For all the conversational preferences except GRT and SER, *p* > 0.05. Hence, the significance of the effect in the cases 1 and 2 becomes of interest. A probable reason for this is that, in almost all the occasions, NI was preferred, and the user gave prominence to the task despite how many people were around. This was the same when the user preferred TLK and CON as well. In such situations, the user gave prominence for relaxation by means of conversation, rather than the task. An example was when the user was in a phone call or a desk activity. In such a situation, user will not prefer to be interacted. Hence, the conversational preference becomes NI. If the user was having a snack, alone, in the living room, he would prefer to have a long conversation and will focus on the conversation without much consideration about performing the task properly. As a whole, conversational preferences at the two ends: NI and “having a friendly conversation” (TLK and CON) had no influence from the living area but middle interaction types (GRT and SER) had. For GRT and SER, where *p* = 0.034 and *p* = 0.046, the null hypothesis could not be accepted. Hence, it can be concluded that there exists a significant difference in the conversational preference for GRT and SER, when the living area changes.

Significant rises and drops in conversational preferences were observed with the change in the number of people around. This is demonstrated in Figure 8. When the overall frequencies of NIs for all the tasks for both occasions are considered, there was a drop in “no interaction” preference when few people were present around the user. One possible reason for this is that a user tend to take a service from the robot, on behalf of all the humans around. However, this drop was not from a significant percentage. The inverse happened with “greeting”; the demand for GR was higher when few people were around the user. The reason for this is the human tendency to hide the desire towards interaction and become inwardly in a social environment. Therefore, people became more introvert with the presence of other humans. The expectancy of service increased when there were few people around. Therefore, a significant increase for SER was observed when the user situation changed from “alone” to “with few people around.” This increase was by 14%. As TLK and CON are rather friendlier types of interaction, these were preferred by the users mostly when they were alone. The percentage differences for these two types of interaction were 28% and 16%. The highest percentage difference for these two occasions was observed in TLK. A possible reason for this is that TLK is the most flexible type of interaction which a user can have without getting disturbed to his/her task. In the meantime, the user will get a chance to have a friendly interaction with the robot, without getting bored by the task or too involved in the task.

From the results shown in Table 3, behavioral changes observed when the user was alone, and when few people were around were analyzed separately. From the first ANOVA test, a *p* value of 1 (≥0.05) and an *F* value of NI could be observed for comparing conversational preferences within each social area: living room, bed room, and the kitchen. Therefore, the fact that “there is a significant difference in the conversational preferences with the social area when the user was performing a task alone” cannot be accepted. In the same way, from the second ANOVA test in Table 3, when few people were around, *p* value of 0.9997 (~1) and an *F* value of 0.00029 (~0). Hence, the fact that “there is a significant difference in conversational preferences when the user was surrounded by a few people in the surrounding” also cannot be accepted. From the two tests, we could observe that there is no significant effect of the type of living area upon conversational preference of a particular user but his task.

According to the two ANOVA tests in Table 5, in both the cases, when the user was alone and was with one/few people around, *F* values (4.442, 21.979) were larger than *F* critical (2.539). Hence, in both these cases, the null hypothesis can be rejected. Hence, the assumption that “there is no significant difference between each type of conversational preference during the selected set of tasks” was declined. Therefore, it can be deduced that the preferences for NI to CON were significantly different when the given tasks were considered. Furthermore, in both the occasions, *p* values (0.035, 7.053E-11) were smaller than the alpha variable (0.05). This also suggests that the individual variables were statistically significant. During “with people” situation, the *F* value (21.979) was significantly larger than the *F* critical (2.539). Hence, the joint effect of all the variables together is larger than that when the user was “alone.”

Another fact observed during the study was that the existence of a significant difference in conversational preferences based on the task. This is examined in the chart in Figure 9. In Figure 9, the frequency of the users who used each type of interaction is plotted against each type of interaction while the user was engaged in the selected task. In all the occasions, the domestic area was the living room, and the user was alone in the environment. Unlike previous experiments, here, we categorized conversational preferences based on the current task of the participant. We recorded the number of participants who go for each conversational preference during the activity. For example, 32% of the total participants preferred SER when they were “reading while being seated.” This is represented by the third (in green) column under “Reading while sitting” in the graph shown in Figure 9. As seen from the chart, there were significant differences in user's conversational preferences when their task changed. For example, few users have chosen NI while resting but many users have chosen NI while making a phone call. In the two occasions, the percentage frequency of users adopted NI was 11% and 76% which reflect a huge difference in adoption of NI during the two activities. As a whole, there was a considerable variation in conversational preferences in the six tasks considered here. People were comfortable with only certain types of interaction when most tasks were considered. This fact was confirmed by the results shown in Figure 9.

## 5. Conclusions and Implications

Continuation of a conversation while perceiving conversational preferences of a user is an important aspect in human-robot interaction. In the paper, findings related to human conversational preferences from a WoZ experiment are presented. Interaction was initiated in the form of a conversation between the robot and the human. The length of a conversation was used as a mediator to monitor the user preference for a short or long interaction with the robot. In this case, the conversational preference was used as a major contributor to perceive human interest and attention towards the robot while some factors in the environment or factors within the user change. According to the current researches, the behavior of humans among acquaintances, their responses will be friendlier in the presence of family or relatives (e.g., a domestic environment) and less friendly in the presence of strangers (e.g., a public space). Therefore, this study can be used to find tendencies of humans in general and to derive those in common encounters.

A teleoperated robot was used to perceive human situation by means of conversational preferences when the above factors were subjected to change. The experiment was intended to reveal the relationship between internal (user-related) and external (environment-related) and conversational preferences of humans. We considered three such factors: user's task, people in the surrounding, and the type of domestic area. During the study, we intended to see if these internal and external factors influence the conversational preference of a person. We considered five conversational preferences: no interaction, greeting, asking for a service, small talk, and long conversation, depending on the length of the conversation. Interesting facts regarding conversational preferences based on the changes related to the user and the surrounding were revealed during the analysis of data. The findings of the study are expected to be used to rebuild modern interaction mechanisms among humans and robots, so that the two conversants (human and robot) are motivated towards a sustaining conversation. Results show that there are considerable effects from factors in the surrounding and the user, upon the conversational preference of a user at that particular time. Moreover, despite age differences, these factors have become prominent in deciding conversational preferences during a particular moment. Furthermore, these findings can be made useful in developing adaptive robotics systems which are expected to be used in social environments.

Although WoZ allowed us to prototype a domestic human-robot scenario, the simulation process was constrained by some realistic situations. As a result, we have implemented only a limited number of factors that affect human conversational preferences in a domestic human-robot scenario. However, the system was capable to explore novel tendencies in human behavior during human-robot interaction and successfully implemented the required conversation skills to make the process of interaction convenient and friendly. Furthermore, we believe that there will be other factors which could be influential in human conversational preferences towards an interaction with a robot. For example, humans are more likely to accept a robot which will look and speak in the way a human does. Hence, patterns in speech, appearance, and personality traits of the robot would also influence the acceptance of a robot. Therefore, evaluation of such facts is important as well. In the future, it is expected to evaluate the personal characteristics of humans towards conversational preferences. Moreover, present robots utilize limited capabilities in comparison to a human. Therefore, the capabilities of the robot will eventually be improved in the future research.

Out of the three aspects: *robot*, *user*, and *environment*, only *user* and *environment* were evaluated in this study. In the future, it is expected to evaluate the *robot* aspect as well, in order to make the human-robot interaction process much more lively and effective.

### 5.1. Implications for Theory

Results suggest that there are factors in the environment and within the user itself, which affect user responses during a certain situation. Therefore, the conceptual design of a robot's intelligence must consider these factors before implementing its task-specific actions.

Findings of the study were based on a limited number of tasks selected from the environment and the user itself. In a real-life scenario, this number will be much higher than the number of factors considered here. Therefore, a maximum number of parameters must be observed from the user and his/her environment before the decision-making process of a robot. Therefore, this could not replicate all parts of the HHI (human-human interaction) into the HRI scenario.

These findings were based on the assumption that people prefer the same rules of interaction with the robot as they do when interacting with humans. There can be certain cultures and social groups in which there are alterations in this fact [38]. Hence, such persons would react to robots in a different manner. In addition, behavior adaptation is as important as behavior monitoring in such a scenario. Several other factors which influence interaction such as the gender, previous experience, and familiarity with the robot were not considered within the context of this experiment.

### 5.2. Implications for Design

Findings suggest that this evaluation offers better means of determining an appropriate conversational preference based on several factors within the user and the environment. As users prefer their robots not to interrupt their usual behavior, the first design guideline suggested from these findings is to respect the preferences of humans by simply following their concerns. These “concerns” can be determined by the factors considered in the study. This “sense” of user situation further acts as an etiquette for the robot to fit well in social environments. This can be presented as the second design guideline for social robots.

The third design guideline is to extract information regarding the situation as much as possible. Considering a higher number of cues from the user and the environment increases the chance of an accurate perception of the situation. To perceive a number of such cues, the robot should acquire visual and auditory sensory information for an adequate duration. This will be the forth design guideline for a situation-aware robot.

## Figures and Tables

**Figure 1:** An example domestic environment is shown. In this scenario, the user is involved in a desk activity in the bed room. In order to understand the whole situation, the robot has to be knowledgeable on three aspects: itself, the user, and the surrounding environment. Factors related to these three aspects are marked as 1,2, and 3, respectively.

**Figure 2:** An application of the two theories: occasion 1 (a), user was working and has no idea about the presence of the robot, (b) notices the presence of the robot as it moves and as a result, the user looks at the robot, and (c) stops the work and gives attention to the robot while it approaches the user.

**Figure 3:** An application of the two theories: occasion 2 (a), user was working and has no idea about the presence of the robot, (b) notices the presence of the robot as it moves and looks at the robot, (c) user averts her gaze and give attention to the work, and (d) engage in the work again.

**Figure 4:** Service Robot platform used in the experiment: MIRob.

**Figure 5:** The nature and the length of conversations determine the “type of conversation” existed at a certain occasion. Here “R” and “H” represent the robot and the human user, respectively.

**Figure 6:** An example scenario during the experiment is shown. (a) The user was in the kitchen, having a drink, (b) the robot approached user and initiated a conversation, and (c) interaction continued.

**Figure 7:** A situation in which the user was having a drink and in the surrounding, there was another human without an interaction with the user. Robot approached the user and initiated a conversation.

**Figure 8:** A stacked graph drawn for the comparison of conversational preferences with the two conditions: when the user is alone and when surrounded by few people. The type of interaction is plotted against the frequency of each type of interaction preferred in above two the occasions.

**Figure 9:** This graph depicts how the users picked up conversational preferences during the selected tasks while the domestic area and people in the surrounding were kept constant. Here, the domestic area was the living room, and the user was alone in the area.

**Table 1:** Some of the tasks selected for the study.

Living area	Task
Living room	Resting while sitting
	Reading while sitting
	Having a snack
	Watching television
	Engaged in a desk activity
	Engaged in a conversation
Bed room	Tidying up
	Resting
	Engaged in a desk activity
Kitchen	Cleaning
	Preparing a meal
	Having breakfast

**Table 2:** A comparison of conversational preferences by the type of interaction when the user was alone and when with few people around.

	Alone	With people around
NI, GRT, SER	64%	79%
TLK, CON	36%	21%

**(a):** 

	Alone			
	Mean	Variance		
Living room	20	107.39
Bedroom	20	127.99
Kitchen	20	286.66

ANOVA test				
	SS	DOF	*F*	*p* value
Between groups	0	2	0	1
Within group	2088.22	12		
Total	2088.22	14		

**(b):** 

	With people around			
	Mean	Variance		
Living room	20	116.73
Bedroom	20	309.39
Kitchen	20	263.53

ANOVA test				
	SS	DOF	*F*	*p* value
Between groups	0.1333	2	0.00029	0.9997
Within group	2756.8	12		
Total	2756.93	14		

**Table 4:** *t*-test for the comparison among each type of interaction when the user was alone and with few people around.

Type of interaction	*T* scores	Alone	With people
NI	Mean	20.67	22.33
	Variance	210.33	16.33
	Dof	2	
	*p*	0.852	
	*t*	4.302	
GRT	Mean	8	12.67
	Variance	7	16.33
	*p*	0.034	
	*t*	4.302	
SER	Mean	35.33	44.33
	Variance	82.33	54.33
	*p*	0.046	
	*t*	4.302	
TLK	Mean	21.67	11.67
	Variance	100.33	9.33
	*p*	0.131	
	*t*	4.302	
CON	Mean	14	8.67
	Variance	9	8.33
	*p*	0.246	
	*t*	4.302	

**(a):** 

	Alone			
Groups	Mean	Variance		
NI	24.32	516.63
GRT	8.56	27.67
SER	32.88	317.20
TLK	20.95	256.49
CON	13.29	102.87

ANOVA test				
	SS	DOF	*F*	*p* value
Between groups	4338.20	4	4.442	0.0035
Within groups	13429.51	55		
Total	17767.71	59		

**(b):** 

	With people around			
Groups	Mean	Variance		
NI	23.20	162.64
GRT	13.29	65.69
SER	42.34	193.02
TLK	11.49	25.40
CON	9.68	53.73

ANOVA test				
	SS	DOF	*F*	*p* value
Between groups	8800.10	4	21.979	7.053E-11
Within groups	5505.23	55		
Total	14305.33	59		

## Data Availability

The data used to support the findings of this study may be released upon application to the corresponding author, Chapa Sirithunge, who can be contacted at ra-chapa@uom.lk.
